The article "Consumption Structure Optimization Strategy for Scenic Spots Using the Deep Learning Model under Digital Economy" was retracted in 2023. Reasons: signs of a paper mill; suspected computer-generated content; unreliable results or conclusions; concerns about the data.

# Consumption Structure Optimization Strategy for Scenic Spots Using the Deep Learning Model under Digital Economy

**DOI:** 10.1155/2022/3029528

**Published:** 2022-08-03

**Authors:** Yi Wang, Na Li, Xiaoe Qu

**Affiliations:** ^1^School of Economics and Finance, Xi'an Jiaotong University, Xi'an 710000, China; ^2^School of Animal Science and Technology, Northwest A and F University, Xianyang 712100, China

## Abstract

The purpose is to find out the problems existing in the consumption economy structure of the scenic spots and to promote the rationalization of the consumption economy of the scenic spots. Based on the analysis of the applicability of the backpropagation neural network (BPNN) model, it uses BPNN to analyze the economic development level of Overseas Chinese Town East (OCT East). Firstly, the weight of each index is determined by the Analytic Hierarchy Process (AHP), and the expected value of the comprehensive evaluation is obtained. Secondly, to ensure the validity of the evaluation model for the development level of the tourism complex, the BPNN model is trained and tested to enable it to be applied to the evaluation of the economic development level of OCT East. The development level of OCT East from 2012 to 2021 is divided into three stages: high, higher, and lower. The development characteristics and existing problems of the OCT East are analyzed, and the optimization strategy of the consumption economy of the scenic spots is put forward in a targeted manner. The research results manifest, that from 2012 to 2021, the development level index of OCT East increased from 0.2457 to 0.5304, and it was in a state of steady growth. In 2019, the development level index reached 0.6497, and it was upgraded to “high-level,” but the average development level index of OCT East was only 0.5662, and there was a lot of room for improvement. According to the divided evaluation indicators, the development level of OCT East is evaluated. In 2012, the development level was low. From 2013 to 2018, it was at a high level, and from 2019 to 2021, it was a high level of development. By studying the Tourism Consumption Structure (TCS) of scenic spots in the OCT East, the research method of the consumption economic structure has been expanded. Therefore, it not only provides a reference for optimizing the consumption of scenic spots, but also contributes to the progress of the social tourism economy.

## 1. Introduction

With the rapid development of the world economy, tourism has gradually become a critical regional economic determinant, and tourism consumption has also become the powerhouse of national economic expansion. As an important indicator to measure tourists' consumption, Tourism Consumption Structure (TCS) reflects how much of tourists' consumption demand has been met, and the development characteristics and laws of consumption structure reflect the profound connotation of TCS [1,2]. Meanwhile, diversified and complex tourism demand determines the systematicness and comprehensiveness of tourism destination development. Adjusting industrial tourism structure is a way to realize tourism destination sustainable development (SD). Since the concept of the tourism complex is put forward, its popularity has sprung up, and the construction volume is rising enormously. However, the current tourism development still has problems, such as blindness, uncoordinated industries in tourism destinations, and lack of characteristics of core attractions, which has caused a tremendous waste of social resources [3–5].

Foreign research on consumption structure has seen an earlier start. At the end of the seventeenth century, George King studied the consumption of the working class. Then, Marx and Engels studied consumer goods and classified the means of living and the preliminary consumption structure research. The concept of consumption structure was first put forward by Edward, who classified and analyzed the household consumption of different classes [6]. Engel's law proposed by German economist Engel was a fundamental consumption structure law. He believed that the proportion of food expenditure would continue to shrink with household income increase. In particular, the ratio of food in total household expenditure was termed the Engel coefficient. The smaller its value was, the more reasonable the household consumption structure was [7,8]. In terms of the research method of consumption structure, the British scientist Stone proposed the Large Eddy Simulation (LES) model to study and analyze the consumption law, which had not seen wide applications due to its limitations. Then, the economist Lluch built the Extended Linear Expenditure System (ELES) to make up for the shortcomings of the LES model [9].

By consulting relevant literature, it can be found that the current research mainly focuses on the discussion of the dynamic mechanism and development model of the tourism complex. The research methods are mainly based on various qualitative researches with consumers as the class, and there are relatively few researches on tourism complexes through quantitative models. On the basis of Maslow's hierarchy of needs (MHoN) and consumption structure optimization strategy, the backpropagation neural network (BPNN) model is constructed. The development level and related influence of the tourism complex of OCT East and its various subsystems are analyzed, and its countermeasures for sustainable development are put forward.

## 2. Theoretical Basis and Model Construction

### 2.1. Theoretical Basis

#### 2.1.1. Maslow's Hierarchy of Needs (MHoN)

American psychologist Maslow classifies human needs as low-level (instinctive) and high-level (advanced) needs and states that their low-level demand will gradually weaken as they age. In comparison, advanced needs might constantly appear and grow with chronological and psychological development [10,11]. The subsets of low-level needs can cover physiological, safety, sense of belonging, and needs to love and be loved. The high-level need can be further divided into the need to be respected and self-realization.  Figure 1 classifies the human needs in detail.

People's desire for different needs might vary substantially according to their development stage. Maslow believes that the hierarchy of the five human needs (Figure 1) gradually rises pyramidically, is not completely fixed, and permeates and overlaps. Several kinds of needs might coexist in an individual, of which one demand plays a leading role in human behavior mode. Then, the incentive mainly comes from the unsatisfied demand that gets less stimulative once satisfied [12].

Demand is the direct stimulus and fundamental source of consumption. Only diversified consumption objects can meet the five levels of human needs. However, many factors often restrict the demand for consumption transformation, making it difficult to realize people's actual needs. In that case, people will choose first to meet their low-level needs through basic consumption and then gradually carry out high-level consumption to meet the high-level needs, thus forming the consumption structure dynamics from single to complex. With the development of human society and improved life quality, all kinds of consumption structures will also show a certain law of change driven by demand. In particular, the proportion of material goods and subsistence consumption will gradually decrease in the TCS. In contrast, the proportion of spiritual materials, such enjoyment consumption as shopping and entertainment, will increase progressively [13].

#### 2.1.2. TCS Optimization Theory

Many factors, such as consumer composition and consumption preference, socioeconomic environment, and product supply structure, will affect the consumption structure in actual economic operations. Therefore, consumption structure optimization is the rationalization process, gradually changing from an unreasonable state to an appropriate state through the proper consumption adjustment structure. In this process, certain principles need to be followed. Firstly, the consumption structure optimization should adapt to the development level of social productivity and coordinate with the economic development and social and natural environment. Secondly, the top priority is to meet consumers' multidimensional and diversified needs. The consumption structure optimization should realize the harmonious coexistence between man, environment, and society and promote economic development. It is necessary to comply with the general law of consumption development, constantly meet consumers' demand for enjoyment, and improve personal and consumption quality [14].

Every tourism consumption development will eventually form a unique TCS to reflect the development level of regional tourism better. Macro factors (such as product quality and structure of tourism destination) and micro factors (such as tourists' income level and preferences) will positively impact the TCS of a region. The product supply and tourism industrial structure play a predominant role. Whether the product quality meets the needs of tourists, whether the content structure is balanced, and whether the development of production departments is coordinated are the determinant in the consumption structure rationalization and the tourism consumption level. Therefore, the study of TCS is conducive to establishing a diversified product system and reasonable content production structure to rationalize TCS.

### 2.2. Principle of BPNN

BPNN features the input, output, and hidden layer. The model implementation is based on a backpropagation algorithm. Thus, it inputs the data into the network structure and outputs the results after three-level processing. Nodes of each level are made sure to be independent of each other in the forward propagation, and different levels can only affect the nodes of the forward or backward section [15–18]. When the expected error and output result exceed the acceptable range, the backpropagation mechanism will be excited, and the error signal will be fed back according to the propagation direction. Then, the error between the expected value and output gets ideal by continuously adjusting the weighted neuron connection.

This paper selects a BPNN structure with three layers and is input with *X*_1_, *X*_2_, *X*_3_,…, *X*_*n*_. The output is an expert comprehensive evaluation structure. Meanwhile, the input and hidden layers contain *n* and *p* neurons, respectively. After sample learning and training, the connection weight between the hidden layer and the input layer is *W*_*ih*_(*i*=1,2,…, *n*; *h*=1,2,…, *p*). The thresholds of hidden layer and output layer nodes are *b*_*h*_(*h*=1,2,…, *p*) and *b*_0_(*o*=1,2,…, *q*), respectively. The connection weight between the output layer and the hidden layer is *W*_*ho*_(*h*=1,2,…, *p*; *o*=1,2,…, *q*). The output layer is a single neuron structure [19,20].  Figure 2 illustrates the specific network structure.

### 2.3. Algorithm Process of BPNN

(1) Forward propagation: this process mainly includes the following three steps. First, the data input of the hidden layer node is determined by
  (1) $$\begin{array}{c} R_{j}=\sum_{i=1}^{n}w_{ij}-\theta_{j},\;\left(j=1,2,\ldots ,p\right). \end{array}$$
(i) In (1), *R*_*j*_ is input data; *θ*_*j*_ is range value of neurons in the hidden layer; *w*_*ij*_ is interaction coefficient between neuron *i* in the input layer and neuron *j* in the hidden layer; and *p* is the number of neuron nodes contained in the hidden layer [21, 22].
Then, the data output from the hidden layer node is calculated by
  (2) $$\begin{array}{c} Z_{j}=f\left(R_{j}\right)\\ =\frac{1}{1+e^{-R_{j}}},\;\left(j=1,2,\ldots ,p\right). \end{array}$$
(i) In (2), *Z*_*j*_ is output data.
Finally, the calculation method of the hidden layer can also calculate the output data of output layer nodes.
(2) Error backpropagation: the variance between the ideal output and the actual output is calculated by (3) to evaluate the error:
  (3) $$\begin{array}{c} e_{i}=\frac{1}{2}{\sum \left(d_{i}-Z_{i}\right)}^{2}. \end{array}$$
In (3): *d*_*i*_ is ideal output result; *Z*_*i*_ is model actual output [23].
(3) Hidden layer's internal coefficient adjustment: during error backpropagation, the internal coefficient is adjusted between nodes at different levels, and the error is observed and compared with a preset range. If the error falls within the range, the trained BPNN model is effective, ending the training process. If the error jumps out of the preset range, the hidden layer's internal coefficient must be adjusted further [24, 25]. First, the input increment of the hidden layer is set by
  (4) $$\begin{array}{c} \Delta w_{jt}=-\alpha \frac{\partial e_{t}}{\partial w_{jt}}\\ =-\alpha \frac{\partial e}{\partial R_{t}}\frac{\partial R_{t}}{\partial w_{jt}}\\ =-\alpha \left(Z_{t}-d_{t}\right)Z_{t}\left(1-Z_{t}\right)y_{t}, \end{array}$$
  (5) $$\begin{array}{c} \Delta \theta_{t}=-\alpha \frac{\partial e_{t}}{\partial \theta }\\ =-\alpha \frac{\partial e_{t}}{\partial R_{t}}\frac{\partial R_{t}}{\partial \theta }\\ =-\alpha \left(Z_{l}-d_{t}\right)y_{t}\left(1-Z_{t}\right). \end{array}$$
(i) In (4) and (5): *α* is constant; Δ*w*_*jt*_ is weight correction; Δ*θ*_*t*_ is threshold correction.
Then, the hidden layer increment will increase according to
  (6) $$\begin{array}{c} \Delta w_{\ddot{\sigma }}=-\beta \frac{\partial e_{i}}{\partial w_{\ddot{\sigma }}}\\ =-\beta \frac{\partial e_{i}}{\partial R_{j}}\frac{\partial R_{j}}{\partial w_{\ddot{\sigma }}}\\ =-\beta \frac{\partial e_{i}}{\partial Z_{j}}\frac{\partial Z_{j}}{\partial R_{j}}\frac{\partial R_{j}}{\partial w_{ij}}\\ =-\beta \frac{\partial e_{i}}{\partial Z_{j}}\left(1-Z_{i}\right)x_{i}, \end{array}$$
  (7) $$\begin{array}{c} \delta_{j}=-\frac{\partial e_{i}}{\partial R_{j}}\\ =-\frac{\partial e_{i}}{\partial Z_{j}}Z_{i}\left(1-Z_{i}\right)\\ =y_{i}\left(1-Z_{i}\right)\sum \delta_{i}w_{ji}. \end{array}$$
Accordingly, (8)–(11) can be obtained:
  (8) $$\begin{array}{c} \Delta w_{i}=\beta \delta_{i}x_{i}, \end{array}$$
  (9) $$\begin{array}{c} \Delta \theta_{j}=\beta \delta_{j}, \end{array}$$
  (10) $$\begin{array}{c} w_{ij}^{\prime }=w_{ij}+\Delta w_{ij}, \end{array}$$
  (11) $$\begin{array}{c} \theta_{j}^{\prime }=\theta_{j}+\Delta \theta_{j}. \end{array}$$
(i) Next, the model parameters are iteratively updated with the new process coefficient using the above equations until the final model error meets the preset accuracy range and the training process terminates.
The BPNN comprehensive evaluation mainly includes the following four steps. Step 1 sets the initialization parameters of the model, such as threshold, initial weight, and maximum training times. Step 2 obtains the model input by normalizing the data values of each evaluation index. Step 3 adjusts the neuron parameters according to the error between the actual and expected output, continues the iterative calculation until the obtained parameters meet the preset conditions, and ends the training process [26].  Figure 3 specifies the algorithm flow.
(4) Implementation of BPNN: according to the constructed evaluation system, this section builds a BPNN with 12 indexes. Each parameter in the input layer corresponds to each index in the neural network, so the number of nodes in the input layer is 12 [27]. Since the ultimate purpose of building the BPNN model is to measure the development level of the tourism complex, the output layer node is the comprehensive evaluation value.  Figure 4 demonstrates the implementation of the network model.

The BPNN training process will be significantly affected by the number of hidden layer nodes. Thus, the three most commonly used methods are selected to determine the number ofhidden layernodes, as expressed by (12)–(14):

(12) $$\begin{array}{c} \sum C_{n_{i}}^{i}>k. \end{array}$$

In (12), *k* is sample number; *k* is hidden layer node number; *i* is input node number; If *i* < *n*_*i*_, then *C*_*n*_*i*__^*i*^=0.

(13) $$\begin{array}{c} n{\;}^{\prime }=\sqrt{n+m}+a, \end{array}$$

(14) $$\begin{array}{c} n{\;}^{\prime }={\text{log}}_{2}^{\prime \prime }. \end{array}$$

In (13) and (14), *n*, *m* are the numbers of input and output nodes; *a* is constant (between 1 and 10).

Then, the number of hidden layer nodes is calculated by the above equations to between 5 and 15.

### 2.4. Data Normalization

The selected network learning sample is the comprehensive evaluation value of the development level of each evaluation index in OCT East from 2011 to 2020 and the normalized data. As an early tourism complex in China, the development of OCT East is relatively complete and has strong market influence. The model adopted by OCT East in the development of tourism complexes across the country is representative to a certain extent. To verify the comprehensive evaluation system of the development level of the tourism complex, it takes the OCT East as an example and conducts a comprehensive evaluation and analysis of its development level, thereby revealing the changing characteristics of the OCT East. The research data are mainly from the data reports of related companies in OCT East, and the final results are obtained through research analysis and the following data processing operations.

Since the dimensions of each indicator are different, they cannot be compared. Hence, before the network model training, the indicator data is processed according to the “ Max − Min ” standardization method. The specific calculation method is exhibited in (15) and (16):

(15) $$\begin{array}{c} y_{ij}=\frac{\left(X_{ij}-X_{\text{min}}\right)}{\left(X_{\text{max}}-X_{\text{min}}\right)}, \end{array}$$

where *X*_*ij*_ refers to the original value of the indicator *j* in the sample *i*; *X*_max_ stands for the maximum value of the indicator; *X*_min_ indicates the minimum value of the indicator; *X* denotes positive indicator.

(16) $$\begin{array}{c} y_{ij}=\frac{\left(X_{\text{max}}-X_{ij}\right)}{\left(X_{\text{max}}-X_{\text{min}}\right)}. \end{array}$$

*X* means negative index.

## 3. Experimental Results and Countermeasures

### 3.1. Data Normalization Results

The quantitative indicators of the tourism complex development are obtained from the credit rating announcement of Shenzhen OCT and the annual report of the Holding Co., Ltd., and the brand awareness and quality of the scenic theme spots are quantified through fuzzy theory.  Figure 5 draws the original data of the comprehensive evaluation indicators.

Then, Figure 6 plots the normalized data of the comprehensive evaluation indicators in Figure 5.

### 3.2. BPNN Model Training

#### 3.2.1. Determine the Ideal Output of the Sample

The BPNN model will be trained to produce results as close to the ideal output as possible. Then, this section employs Analytical Hierarchy Process (AHP) method to determine the weight of the development indicators. Accordingly, the final comprehensive evaluation indicator weight of the tourism complex is obtained, as listed in Table 1.

Figure 7 illuminates the hierarchy of level 4 indicators.

The indicator weights determined by the AHP method are weighted and summed with the standardized indicator data, that is, the overall evaluation score *P*=*Ci∗Wi*, *Ci*, *Wi* are the scores and weights of individual indicators. Finally, the expected output of the development level of the tourism complex is revealed in Figure 8.

#### 3.2.2. Simulation Results of BPNN

The BPNN training process involves a large number of data iterations. At the same time, it requires high calculation accuracy and thus certain complexity. Then, this section employs the MATLAB R2014a programming environment to ensure the rationality and scientificity of the results and improve the operation speed so that the command input of the BPNN toolkit is simple and easy to understand.

In Section 2.3, the basic parameters of the network model have been determined. Then, the training parameters will be set. The test samples are the comprehensive evaluation values in 2012 and 2021, and the learning and training samples are the comprehensive evaluation results and indicator evaluation values of OCT East from 2013 to 2020. Suppose the trained network model can adapt to both test and learning (training) samples. In that case, it shows that the network model can better evaluate and predict the development level of the OCT tourism complex in the OCT East.

The normalized input data fall between [0,1]. The functional characteristics of training functions vary. This section uses trainlm as the training function, which has high memory requirements and greatly shortens the running time. The tansig function is used as the transfer function to complete the transfer process between each layer in the network model to minimize the error between the training and the expected values. Before training, the expected training error, the displayed interval, and maximum training times are set as 1e-5, 1, and 100, respectively.

The indicator evaluation value from 2013 to 2020 is selected as the training data of the network model, and the model error converges to the preset value at the fourth iteration.  Figure 9 outlines the training curve.

Next, Figure 10 compares the output of the training sample with the expected result.

Subsequently, the trained model needs to be further tested to ensure that it can be used scientifically.  Figure 11 depicts the results of the test samples (evaluation values after normalization from 2012 to 2021).

Figure 11 indicates that the error between the output and the expected result is within the preset range. Hence, the trained network model has strong adaptability. When the evaluation index changes, the tourism complex's development level can be evaluated through BPNN to manage the real-time dynamics of the tourism complex.

### 3.3. Evaluation Results

Table 2 divides the development into six levels to more intuitively judge the development of OCT East from 2012 to 2021: very high, high, relatively high, general, relatively low, and low.

Figure 12 manifests the evaluation results of the development level of Eastern OCT from 2012 to 2021:

As displayed in Figure 12, from 2012 to 2021, the development indicators of OCT East have steadily increased from 0.2457 to 0.5304. In 2019, the development level index reached 0.6497, rising to a “high level.” Yet, the average development level index of OCT East is only 0.5662, so there is a lot of room for progress. Further, the development level of OCT in the East is evaluated by the divided evaluation indicators. The development level in 2012 is low, at a high level from 2013 to 2018, and at a high level from 2019 to 2021.

### 3.4. Consumption Structure Optimization Strategy

According to the above research results, the following optimization strategies are proposed for the consumption of scenic spots to improve the current consumption situation.

#### 3.4.1. Product Portfolio Diversification

Eastern OCT attaches too much importance to constructing entertainment products and sightseeing products in terms of tourism investment structure. Still, it does not develop special tourism projects, such as health tourism, study tourism, and leisure vacation tourism, resulting in the lack of rationality of the tourism structure of ECT East. Meanwhile, there is also a need to strengthen the coordination of comprehensive service facilities and scenic spots in Shenzhen. The western region gathers large tourist attractions, such as the Window of the World, the Chinese Folk Culture Village, and Splendid China. In contrast, the natural scenery in the eastern region has not been developed. Shenzhen lacks specific strength in developing its advantageous tourism resources as a coastal city.

The product competitiveness can be improved through the combination of products, which should comply with the market orientation and meet the needs of tourists. There is a need to innovate products and services further to improve the product attractiveness and stimulate tourists' purchase desire. On the other hand, marketing strategies should attract tourists through reasonable publicity and increase investment in product form, quality, and after-sales to improve the quality of products. With the development of the experience economy, tourists do not buy products completely out of life needs, but more often out of emotional needs or pursue products consistent with their ideas.

#### 3.4.2. Strengthen Hotel Construction to Meet the Needs of Tourists

As an essential part of tourism development, the healthy development of the accommodation sector plays a vital role in optimizing tourism consumption economic structure in scenic spots. The accommodation industry combines intangible goods with tangible goods. From such a perspective, the following improvement strategies can be put forward: first, the types of hotel services are diversified, which can meet various tourists' needs, such as family tourism, vacation, and tourist meetings. Second, there is a need to manage and improve homestays and hotels' online information so that tourists can have a comprehensive understanding of accommodation information. Third, it is imperative to strictly regulate the evaluation standards of star hotels and provide services and facilities with the same star standards to ensure the health and safety of the accommodation environment.

#### 3.4.3. Build a Diversified Profit Model

OCT East's per capita tourism consumption level is growing slowly, and the market development is stagnant. Therefore, in terms of income model, it is necessary to thoroughly learn from the advanced management experience of scenic spot tourism domestically and globally, promote the growth of income, and actively guide the consumption trend of tourists through supporting tourism management services, such as hotels, catering, and shopping. Thus, the added value can be maximized.

There is a large gap between the income of tourism real estate and that of other tourism enterprises in TOI of OCT East. The operating income mainly depends on real estate enterprises, resulting in a substantial income imbalance. At the initial stage of development, the development model of “tourism + real estate” is conducive to the rapid return of funds. Still, it also leads to problems, such as insufficient power for SD. Hence, it is necessary to rationalize the profit model design of tourism reception enterprises to promote the SD of scenic spot tourism. OCT East should build the following profit models as soon as possible: project appreciation profit, brand benefit, tourism operation profit, and sales profit. Then, it can effectively reduce the project investment risk, ensure the rapid return of project funds, and realize the appreciation of tangible and intangible assets. The above four profit models promote and influence each other that it would be possible to maximize the TOI of the project.

#### 3.4.4. Strengthen Publicity Employing Information Platform

For popularity concerns, modern network platforms can be used to publicize tourism products and resources. It is necessary to improve the tourism consumption of scenic spots and carry out effective marketing according to the market characteristics. At present, the main marketing methods can be summarized as follows:

- Written materials and promotional videos related to scenic spot tourism: they are publicized through large websites, such as Netease, Sina, or TV media.
- Official account of scenic spots in various provinces.

Then, local tourist attractions and related tourism videos can be uploaded to introduce the tourist resources, unique products, and traditional snacks.

#### 3.4.5. Do an Excellent Job of Guarantee

Economic activities are only made possible under government support. The help and guidance of the government can provide a substantial boost for the optimization of the consumption structure of scenic spots. Guarantee work can be started from the following four aspects. (I) Relevant policies can be introduced to optimize the consumption economic structure of scenic spots and standardize consumption activities. Then, there will be laws to follow and rules to make all activities go smoothly. (II) The government should play the role of “Grinding agent” and “Lighthouse,” carrying out macro-control to optimize consumption economic structure, optimize the allocation of resources, cooperate with other economic activities, and achieve fairness and justice. (III) Corresponding reduction and exemption policies can be introduced to reduce tourism expenses and promote optimizing the consumption structure of scenic spots from the policy aspect. (IV) It might improve the TCS through appropriation, ensure capital investment, or support the development of the tourism consumption economy through government publicity platforms.

Service personnel are those who directly serve tourists in tourism activities. Their quality will have an important impact on tourists' feelings and greatly affect the long-term development of scenic tourism. Talents are the primary productive force, and high-quality tourism service personnel are conducive to the improvement of tourism quality. However, there is currently a lack of tourism professionals. Therefore, it is necessary to strengthen the training of tourist service personnel in scenic spots, improve the professional awareness and service level of service personnel such as accommodation, transportation, and catering, and train foreign language tour guides to deal with the language barrier of foreign tourists. Meanwhile, talents in the service field can be introduced from other regions, so that the quality of service personnel can be effectively improved. From the perspective of long-term development, the following two points still need to be done: while ensuring the quality of the training of tourism talents, strengthen the training of tourism professionals, increase the number of tourism colleges, and provide learning opportunities for students who are interested in tourism work. Second, under the existing conditions, practical opportunities for tourism students are provided to enhance their professional skills. Combined with the professional training plan, the training of practical ability is included in the student assessment, and efforts are made for the training of tourism talents. To sum up, the implementation of these strategies first requires the support of the government; second, management and service enterprises need to carry out internal training and optimization of the management system. Finally, enterprises need to carry out corresponding publicity in the scenic spot to improve the popularity.

## 4. Conclusions

As a critical indicator to measure tourists' consumption, consumption structure reflects the realization of tourists' consumption demand, and its development characteristics and laws reflect the deep connotation of TCS. The large-scale construction of tourism complex puts forward higher requirements on technology, ecology, capital and resources. Comprehensive evaluation of the development level of tourism complexes and exploration of its scientific development path are of great significance to regional tourism and the overall development of the region. From this, BPNN is used to analyze the economic development level of OCT East. First, the weight of each index is determined by AHP, and the expected value of comprehensive evaluation is obtained. Then, to ensure the validity of the evaluation model of the development level of the tourism complex, the BNN model is trained and tested so that it can be applied to the economic development level of OCT East in the evaluation. The research results illustrate that the development level of OCT East from 2009 to 2018 is divided into three stages: high, higher, and lower. Its development characteristics and existing problems are analyzed, and the consumption economy optimization strategy of the scenic spots is proposed. In the process of research, BPNN technology is selected as the main research method. Although the content has been comprehensively analyzed, the current research method can analyze the scene is too small, and the representativeness of the results is relatively low. Therefore, it is necessary to deeply optimize the BPNN technology in the future to improve the research effect.

## Figures and Tables

**Figure 1:** MHoN.

**Figure 2:** BPNN structure.

**Figure 3:** Algorithm flow chart.

**Figure 4:** Implementation of BPNN.

**Figure 5:** Original data of comprehensive evaluation indicators of tourism complex. (a) Scale and quality of scenic theme spots. (b) Brand awareness.

**Figure 6:** Normalized dimensionless data. (a) X1—X6; (b) X7—X12.

**Figure 7:** Four hierarchy indicator layer weight. (a) Single hierarchy sorting. (b) Overall hierarchy sorting.

**Figure 8:** Expected output.

**Figure 9:** Development level training path.

**Figure 10:** Analysis of training sample results.

**Figure 11:** Comparison of output results.

**Figure 12:** Development level of OCT East.

**Table 1:** Weight of comprehensive evaluation indicator of tourism complex.

Primary index	Secondary index	Weight	Tertiary index	Weight	Fourth-level index	Index
The development level of tourism complex	Tourism core attraction subsystem	0.5324	Theme scenic spot	0.8405	The scale of scenic theme spot	X1
			Land use	0.1596	Land use degree	X2
	Tourism reception enterprise subsystem	0.1548	The scale of tourism reception enterprises	0.3756	The scale of tourism and accommodation enterprises	X3
					The scale of tourism catering enterprises	X4
					The scale of tourism shopping enterprises	X7
					The scale of theme tourism real estate	X8
			Operation level of tourism reception enterprises	0.6247	Operating income of tourism and accommodation enterprises	X5
					Income of other tourism reception enterprises	X6
					Theme tourism real estate operation level	X9
			Tourist market scale	0.2820	Total number of tourists	X10
					Per capita tourism consumption	X11
					Total operating income (IOI)	X12

**Table 2:** Evaluating indicator.

Development level	Output result *b*
Low	0.1 < *b* ≤ 0.2
Relatively low	0.2 < *b* ≤ 0.3
General	0.3 < *b* ≤ 0.4
Relatively high	0.4 < *b* ≤ 0.6
High	0.6 < *b* ≤ 0.8
Very high	0.8 < *b* ≤ 1.0

## Data Availability

All data can be obtained from the corresponding author upon request.
